The article "Numerical Simulation of MHD Couette Flow of a Fuzzy Nanofluid through an Inclined Channel with Thermal Radiation Effect" was published in 2021. Journal: Comput Intell Neurosci.

# Numerical Simulation of MHD Couette Flow of a Fuzzy Nanofluid through an Inclined Channel with Thermal Radiation Effect

**DOI:** 10.1155/2021/6608684

**Published:** 2021-10-31

**Authors:** Imran Siddique, Rana Muhammad Zulqarnain, Muhammad Nadeem, Fahd Jarad

**Affiliations:** ^1^Department of Mathematics, University of Management and Technology, Lahore 54770, Pakistan; ^2^Department of Mathematics, University of Management and Technology, Lahore, Sialkot Campus, Pakistan; ^3^Department of Mathematics, Cankaya University, Etimesgut, Ankara, Turkey; ^4^Department of Medical Research, China Medical University Hospital, China Medical University, Taichung, Taiwan

## Abstract

The present study especially concerns the investigation of the Couette flow and heat transfer with thermal radiation through an inclined channel. Single-wall carbon nanotube (SWCNT) and multiple-wall carbon nanotube (MWCNT) are nanoparticles embedded in the host fluid. The dimensionless highly nonlinear differential equations (DEs) are solved via numerical scheme bvp4c. The effects of the physical parameters on heat transfer are presented in the form of graphs. The results demonstrate that the heat transfer is enhanced by using solid particle frictions (SWCNT and MWCNT). The large estimation of a magnetic parameter declines the velocity component. The current and existing results with their comparisons are shown in the tabular form for the validation of our code. The current results are in good agreement with their existing results. Generally, fuzziness or uncertainty is inherent in modeling, analysis, and experimentation. Due to the uncertain environmental conditions, fuzziness broadly exists in various engineering heat transfer problems. In this work, the nanoparticles' volume fraction of the SWCNT and MWCNT is taken as uncertain parameters in terms of triangular fuzzy numbers (TFNs). The TFNs are controlled by the *α* − cut which has less computational effort for analyzing the fuzziness or uncertainties. Also, a comparison between the SWCNT and MWCNT through the membership function and the variability of the uncertainty is studied.

## 1. Introduction

The study of the flow of third-grade fluids [1–3] over an inclined channel is an important application in engineering, science, and technology. Some of these applications can be found in materials manufactured by the extraction procedure particularly in polymer processing, the flow of synovial fluid in human joints, geological flows inside the Earth's mantle, microfluids, drilling of oil and gas wells, etc. In fluid dynamics, the study of fundamental flow, namely, Couette flows to attract the researchers by several non-Newtonian fluids because of their uses in the technology and engineering industry. The unidirectional flow is used in polymer engineering such as die flow, injection molding, extrusion, plastic forming, continuous casting, and asthenosphere flows [4–7]. Magnetohydrodynamics (MHD) deals with the study of the motion of electrical fluids in the presence of a magnetic field. MHD flow has significant importance applications in the inclined channel such as geophysical, astrophysical, metallurgical processing, MHD generators, pumps, geothermal reservoirs, polymer technology, and mineral industries. MHD fluid uses as a lubricant to stop the unexpected variation of fluid viscosity with temperature under certain norms. Thermal radiation is a process by which energy, in the form of electromagnetic radiation, is emitted by a heated surface in all directions and travels directly to its point of absorption at the speed of light; thermal radiation does not require an intervening medium to carry it. Thermal radiation plays an important role in science and technology, such as the furnace design, glass production, ship compressors, space vehicles, plasma physics, propulsion systems, spacecraft, flow structure of atomic plants, internal combustion engines, combustion processes, gas turbines, solar radiations, and solar power technology. Kamran and Siddique [8] calculated the analytical solutions for MHD flow between infinite parallel plates. Siddiqui et al. [9] calculated the deliberated flow of a third-grade fluid between two inclined parallel plates with heat transfer using the homotopy perturbation method (HPM). Aiyesimi et al. [10] studied the MHD Couette flow and Poiseuille flow problems using the homotopy perturbation method (HPM) and perturbation method (PM). They examined that both methods have the same solutions. Later on, Aiyesimi et al. [11] studied the solution of MHD Couette flow and Poiseuille flow problems of the temperature and velocity profile utilizing the perturbation method (PM). Yusuf et al. [12] studied the Couette flow with the effect of Soret, Dufour, and thermal radiation using the modified domain decomposition method (MADM) in an inclined channel. Okedayo et al. [13] used the MADM to study the viscous dissipation, Joule heating, and MHD flow of a third-grade fluid in an inclined channel. Farooq et al. [14] used the PM to study the Poiseuille flow of a couple of stress fluids with variable viscosity between two parallel inclined heated plates. Zeeshan et al. [15] studied the impact of variable thermal conductivity, heat generation, heat flux, and inclined uniform magnetic field on Poiseuille flow employing the homotopy analysis method (HAM). In this way, there are large kinds of literature about MHD and thermal radiation such as [16–23].

The article "Numerical Simulation of MHD Couette Flow of a Fuzzy Nanofluid through an Inclined Channel with Thermal Radiation Effect" was published in 2021. Journal: Comput Intell Neurosci.

Heat transfer is important in industrial areas to launch transportation of energy in the system. Heat transfer is an essential task due to the requirement for energy in the world. In recent years, nanofluids have great attention because of their large-scale usage in industries. There are many applications of nanofluids in science and engineering, such as heat exchangers, solar cells, cooling of electronic equipment, solar water heaters, cooling of diesel-electric generators, nuclear reactors, cooling, and heating in buildings. The range of nanoscale particles is 1–100 nm, which benefits to increase the thermophysical properties of the nanofluid. Due to an increase in energy prices, the management of heat transfer is a vital role in energy systems. The nanofluids are the mixture of solid-liquid which contain nanoparticles for enhancing the heat transfer, investigated by Choi and Eastman [24]. The performance of nanoparticles in a heat transfer mechanism is better than the base fluid; the reason is that the suspended ultrafine particles increase the thermal conductivity of the mixture and raise their competency of energy transfer. Numerous literature studies [25–27] disclose the low volume fractions (1%–20% volume) for better performance of thermal conductivity of the suspensions; we can take more than 20% nanoparticles' concentrations. Carbon nanotubes (CNTs) are cylindrical shape materials made of graphene. There are two types of CNTs, SWCNT and MWCNT, which are used in this work. As compared to other nanomaterials, SWCNT and MWCNT are of great importance for scholars due to their significant thermal conductivities, bent without any damage, and mechanical power. Saqib et al. [28] studied natural convection flow using carboxymethyl cellulose (CMS) as a base fluid and CNTs as hybrid nanofluids between two vertical parallel plates. For the exact solution, the Caputo–Fabrizio fractional derivative with the Laplace transform method is used. Hatami and Ganji [29] discussed the natural convection flow of sodium alginate (SA) as a base fluid and copper (Cu) and silver (Ag) as a nanofluid between two vertical parallel plates using the differential transform method (DTM). Khan et al. [30] studied the Navier slip boundary conditions for heat transfer using CNTs. Noreen et al. [31] studied the velocity slips and thermal analysis on MHD peristaltic flow in an asymmetric channel using CNTs. Ebaid and Al Sharif [32] deliberated the effect of MHD on nanofluids' motion using CNTs and enhanced the heat transfer rate. The flow and heat transport of a special kind of second-grade hybrid Al_2_O_3_+Cu/H_2_O nanofluid over a permeable stretching/shrinking sheet was addressed by Roy and Pop [33].

The article "Numerical Simulation of MHD Couette Flow of a Fuzzy Nanofluid through an Inclined Channel with Thermal Radiation Effect" was published in 2021. Journal: Comput Intell Neurosci.

The flow of fluids with heat transfer is essential in science and engineering. After controlling the physical quantities like chemical diffusion, magnetic effect, volume friction of nanoparticles, and heat transmission, the fluid models are transformed into linear and nonlinear DEs. After governing these physical problems, they are converted into linear or nonlinear DEs. In general, the physical problems with involved geometry, coefficients, parameters, and initial and boundary conditions greatly affect the solution of DEs. Then, the coefficients, parameters, and initial and boundary conditions are not crisp due to the mechanical defect, experimental error, and measurement error. So, in this situation, fuzzy set theory is a powerful tool for a better understanding of the considered phenomena, and it is more accurate than assuming the crisp or classical physical problems. To be more specific, FDEs play a significant role in reducing uncertainity and providing a correct approach to characterise a physical issue with unknown parameters, initial and boundary conditions.

In 1965, Zadeh [34] presented the fuzzy set theory (FST). FST is a very valuable tool to define the situation in which information is imprecise, vague, or uncertain. FST is completely defined by its membership function or belongingness, and the membership function describes each element of the universe of discourse by a number from the [0, 1] interval. On the contrary, the degree of nonbelongingness is a complement to “one” of the membership degree or belongingness. Fuzzy number (FN) can be expected as a function whose range is specified from zero to one. Every numerical value in the range is allocated a definite grade of the membership function where zero signifies the minimum possible grade and one is the maximum possible grade. Arithmetic operations on FNs were developed by Dubois and Prade [35]. Different types of FNs can be categories in triangular, trapezoidal, and Gaussian fuzzy numbers. Here, we consider TFNs for the sake of completeness. Also, many scholars have applied FST to obtain well-known results in the field of commerce and science [36–46].

The information of dynamical systems modeled by partial or ordinary differential equations is commonly incomplete, vague, or uncertain, while FDEs represent a proper way to model the dynamical systems under vagueness or uncertainty. This impreciseness or vagueness can be defined mathematically using FNs or TFNs. In recent years, there have been many studies revolving around the concept of FDEs. Seikala [47] introduced the fuzzy differentiability concept. Later on, Kaleva [48] presented fuzzy differentiation and integration. Kandel and Byatt [49] introduced the FDEs in 1987. Buckley et al. [50] used two methods' extension principle and FNs for the solution of FDEs. Gasilov et al. [51] studied the system of FDEs with the TFNs. Salahshour et al. [52] studied the fuzzy logistic equation and alley effect using FDEs with the help of TFNs. Biswal et al. [53] studied the natural convection of nanofluid flow between two parallel plates using the HPM in a fuzzy environment. The volume fraction of nanoparticles is considered as the TFN and also shows that the fuzzy result is better than a crisp result. Borah et al. [54] discussed the MHD flow of second-grade fluids in a fuzzy environment using fractional derivatives Atangana–Baleanu and Caputo–Fabrizio. The nondimensional governing equations are converted into fuzzified governing equations with the help of the Zadeh extension principle and triangular fuzzy number. MHD and ohmic heating on the third-grade fluid in an inclined channel in a fuzzy environment was investigated by Nadeem et al. [55]. To discuss the uncertainty, the triangle membership function was used.

The article "Numerical Simulation of MHD Couette Flow of a Fuzzy Nanofluid through an Inclined Channel with Thermal Radiation Effect" was published in 2021. Journal: Comput Intell Neurosci.

In the literature review, it scrutinized that there is no such study that has been accounted in an MHD Couette flow with pure water as the base fluid and CNTs (SWCNTs and MWCNTs) as nanoparticles through the inclined heated channel in the presence of thermal radiation. The governing nonlinear coupled ordinary differential equations are solved by numerical scheme bvp4c. Furthermore, after checking the accuracy of bvp4c, the results of existing works in the literature are compared. The nanoparticles' volume fraction performs the main role in the enhancement of heat transfer and thermophysical properties. The particular applications of nanoparticles are in solar water heating, engine cooling, cooling of transformer oil, cooling of the radiator, cooling in machining, and defense. Some researchers take nanoparticles' volume fraction 0 to 4% for the enhancement of heat transfer. However, from different sources [25–27], we can take nanoparticles' volume fraction more than 20% for better performance of heat transfer. So, the volume fraction of nanoparticles (SWCNTs and MWCNTs) is taken as a fuzzy number or uncertain because it depends on the added nanoparticle volume or dimensions of particles or the shape of particles of the fluid. In this respect, volume fraction has been taken as an uncertain parameter in terms of fuzzy numbers in the present study. To handle this problem in a fuzzy environment, FDEs and the triangular fuzzy plot with the *α* − cut approach were used. Also, the comparison of SWCNTs and MWCNTs is discussed through triangular fuzzy plots.

The article "Numerical Simulation of MHD Couette Flow of a Fuzzy Nanofluid through an Inclined Channel with Thermal Radiation Effect" was published in 2021. Journal: Comput Intell Neurosci.

## 2. Preliminaries

In this section, some basic notations and definitions are used.

**Definition 1 (see [34]).**

Fuzzy set is defined as a set of ordered pairs such that $\tilde{U}=\left\{\left(y,\mu_{\tilde{U}}\left(y\right)\right):y\in X,\mu_{\tilde{U}}\left(y\right)\in \left[0,1\right]\right\}$, where *X* is the universal set and $\mu_{\tilde{U}}\left(y\right)$ is the membership function of $\tilde{U}$ and mapping defined as $\mu_{\tilde{U}}\left(y\right):X⟶\left[0,1\right]$.

**Definition 2 (see [35]).**

The *α* − levelor *α* − cut of a fuzzy set $\tilde{U}$ is a crisp set *U*_*α*_ and defined by $U_{\alpha }=\left\{y/\mu_{\tilde{U}}\left(y\right)\geq \alpha \right\}$, where 0 ≤ *α* ≤ 1.

**Definition 3 (see [35, 55]).**

Let $\tilde{U}=\left(a_{1},a_{2},a_{3}\right)$ with membership function $\mu_{\tilde{U}}\left(y\right)$ be called a membership function of the TFN if

(1) $$\begin{array}{c} \mu_{\tilde{U}}\left(y\right)=\left\{\begin{array}{cc} \frac{a_{1}-y}{a_{1}-a_{2}}, & \text{for }y\in \left[a_{1},a_{2}\right],\\ \frac{a_{3}-y}{a_{3}-a_{2}}, & \text{for }y\in \left[a_{2},a_{3}\right],\\ 0, & \text{otherwise.} \end{array}\right) \end{array}$$

Membership functions allow us to graphically represent a fuzzy set. The *x*-axis signifies the universe of discourse, while the *y*-axis signifies the degrees of membership in the [0, 1] interval. The TFNs with peak (or center) a_2_, left width a_2_- a_1_ > 0, and right width a_3_-a_2_ > 0 are transformed into the interval numbers through *α*-cut approach, which is written as $\tilde{U}=\left[u_{1}\left(y;\alpha \right),u_{2}\left(y;\alpha \right)\right]=\left[a_{1}+\alpha \left(a_{2}-a_{1}\right),a_{3}-\alpha \left(a_{3}-a_{2}\right)\right]$, where 0 ≤ *α* ≤ 1. A TFN $\tilde{U}=\left(a_{1},a_{2},a_{3}\right)$ and the *α*-cut of the membership function are seen in Figure 1. An arbitrary TFN satisfies the following conditions: (i) *u*_1_(*y*; *α*) is an increasing function on [0, 1]. (ii) *u*_2_(*y*; *α*) is a decreasing function on [0, 1]. (iii) *u*_1_(*y*; *α*) ≤ *u*_2_(*y*; *α*) on [0, 1]. (iv) *u*_1_(*y*; *α*) and *u*_2_(*y*; *α*) are bounded on left continuous and right continuous at [0, 1], respectively. (v) *u*_1_(*y*, *α*)=*u*_2_(*y*, *α*)=*u*(*y*) where *u*(*y*) is a crisp number at *α* − cut=1.

*U*_*α*_ must be a closed interval for every 0 ≤ *α* ≤ 1; also, *α* is called the level of credibility or presumption. Membership function or grade is also named as a grade of possibility or grade of credibility for a given number. Also, Figure 1 describes the membership function of a triangular fuzzy uncertainty. So, the triangular fuzzy uncertainty is defined as *u*_1_(*y*; *α*) (lower bound), *u*(*y*) (most belief value), and *u*_2_(*y*; *α*) (upper bound).

The article "Numerical Simulation of MHD Couette Flow of a Fuzzy Nanofluid through an Inclined Channel with Thermal Radiation Effect" was published in 2021. Journal: Comput Intell Neurosci.

**Definition 4 (see [47, 50, 55]).**

Let *I* be a real interval. A mapping $\tilde{u}:I⟶F$ is called a fuzzy process, defined as $\tilde{u}\left(y;\alpha \right)=\left[u_{1}\left(y;\alpha \right),u_{1}\left(y;\alpha \right)\right],y\in I$ and *α* ∈ [0,1]. The derivative $d\tilde{u}\left(y;\alpha \right)/dy\in F$ of a fuzzy process $\tilde{u}\left(y;\alpha \right)$ is defined by $d\tilde{u}\left(y;\alpha \right)/dy=\left[du_{1}\left(y;\alpha \right)/dy/du_{2}\left(y;\alpha \right)/dy\right]$.

**Definition 5 (see [47, 50, 55]).**

Let $I\subseteq R\text{ and }\tilde{u}$ be a fuzzy-valued function defined on *I*. Let $\tilde{u}\left(y;\alpha \right)=\left[u_{1}\left(y;\alpha \right),u_{2}\left(y;\alpha \right)\right]$ for all *α*-cuts. Assume that *u*_1_(*y*; *α*) and *u*_2_(*y*; *α*) have continuous derivatives or are differentiable, for all *y* ∈ *I* and *α*; then, ${\left[d\tilde{u}\left(y;\alpha \right)/dy\right]}_{\alpha }={\left[du_{1}\left(y;\alpha \right)/dy/du_{2}\left(y;\alpha \right)/dy\right]}_{\alpha }.$ Similarly, we can define higher-order ordinary derivatives in the same way. An FN by an ordered pair of functions ${\left[d\tilde{u}\left(y;\alpha \right)/dy\right]}_{\alpha }$ satisfies the following conditions: (i) *du*_1_(*y*; *α*)/*dy* and *du*_2_(*y*; *α*)/*dy* are continuous on [0, 1]. (ii) *du*_1_(*y*; *α*)/*dy* is an increasing function on [0, 1]. (iii) *du*_2_(*y*; *α*)/*dy* is a decreasing function on [0, 1]. (iv) *du*_1_(*y*; *α*)/*dy* ≤ *du*_2_(*y*; *α*)/*dy* on [0, 1].

## 3. Problem Formulation

Consider the steady incompressible Couette flow of pure water as a base fluid, and SWCNT and MWCNT nanoparticles are added separately in an inclined channel with heat transfer. The distance between two inclined parallel plates is 2*H* with the *x*-axis as the flow direction. The upper plate is moving with constant speed *U*, while the lower plate is fixed. The plates having constant temperatures with the upper plate instantaneously change in temperature *T*_2_ − *T*_1_. An unchanging magnetic field *B*_0_ is applied in the *y*-direction and is expected undisturbed as the induced magnetic field is neglected under the assumption of a small magnetic Reynolds number. Radiative heat flux is considered here. The pressure and ambient air are ignored so that the flow is due to the movement of the upper plate and alone with gravity. The properties of SWCNTs, MWCNTs, and water are given in Table 1.

In the equations, the flow of an incompressible, unidirectional, third-grade fluid with the effects of MHD is given [8–11]:

(2) $$\begin{array}{c} \text{div}V=0, \end{array}$$

(3) $$\begin{array}{c} \rho \frac{dV}{dt}=-\nabla p+\text{div}\hat{S}+J\times B+f\rho , \end{array}$$

(4) $$\begin{array}{c} B=B_{\circ }+b, \end{array}$$

where *ρ* is the constant density, *d*/*dt* is the material derivative, **V** is the velocity vector, *p* is the pressure, *τ*^*∗*^ is the stress tensor, **J** is the electric current density, **B** is the total magnetic field, **B**_∘_ denotes the imposed magnetic field, and **b** represents the induced magnetic field.

(5) $$\begin{array}{c} J=\sigma \left[V\times B+E\right], \end{array}$$

(6) $$\begin{array}{c} \nabla \times B=\mu_{m}J,\\ \nabla \cdot B=0, \end{array}$$

where **E** is the electric field (**E**=0), *μ*_*m*_ is the magnetic permeability, and *σ* is the electrical conductivity.

(7) $$\begin{array}{c} \hat{S}=\mu A_{1}+\alpha_{1}A_{2}+\alpha_{2}A_{1}^{2}+\beta_{1}A_{3}+\beta_{2}\left(A_{2}A_{1}+A_{1}A_{2}\right)+\beta_{3}\left(\text{tr}A_{1}^{2}\right)A_{1}, \end{array}$$

wherein *μ* is the coefficient of viscosity and *α*_1_, *α*_2_, *β*_1_, *β*_2_, and *β*_3_ are material constants. The Rivlin–Ericksen tensors **A**_*n*_ are defined as **A**_∘_=*I* is the identity tensor:

(8) $$\begin{array}{c} A_{n}=\frac{dA_{n-1}}{dt}+A_{n-1}\left(\text{grad}V\right)+{\left(\text{grad}V\right)}^{T}A_{n-1},\;n\geq 1. \end{array}$$

The geometry of the problem is presented in Figure 2.

The article "Numerical Simulation of MHD Couette Flow of a Fuzzy Nanofluid through an Inclined Channel with Thermal Radiation Effect" was published in 2021. Journal: Comput Intell Neurosci.

For radiation, Rosseland approximation is used [16–18]:

(9) $$\begin{array}{c} q_{r}=-\frac{4\sigma^{*}}{3k^{*}}.\frac{\partial T^{4}}{\partial y}, \end{array}$$

where *σ*^*∗*^ is the Stefan–Boltzmann constant, *k*^*∗*^ is the absorption coefficient, and *T*^4^ is the linear temperature function. *T*^4^ is expanded by Taylor series expansion about *T*_*∞*_ as

(10) $$\begin{array}{c} T^{4}=4T_{\infty }^{3}T-3T_{\infty }^{4}. \end{array}$$

Define velocity and temperature profiles for one-dimensional flows as follows [8, 11, 55]:

(11) $$\begin{array}{c} V=\left[\begin{array}{ccc} u\left(y\right) & 0 & 0 \end{array}\right],\theta =\theta \left(y\right). \end{array}$$

Using equations (2)–(6) along with equations (7)–(11),

(12) $$\begin{array}{c} \mu_{nf}\frac{d^{2}V}{dy^{2}}+6\left(\beta_{2}+\beta_{3}\right){\left(\frac{dV}{dy}\right)}^{2}\frac{d^{2}V}{dy^{2}}+g\rho_{nf}\sin\;\gamma -\sigma_{nf}B_{o}^{2}V=0, \end{array}$$

(13) $$\begin{array}{c} k_{nf}\frac{d^{2}T}{dy^{2}}+\mu_{nf}{\left(\frac{dV}{dy}\right)}^{2}+2\left(\beta_{2}+\beta_{3}\right){\left(\frac{dV}{dy}\right)}^{4}-\frac{1}{{\left(\rho c_{p}\right)}_{f}}\frac{dq_{r}}{dy}+\sigma_{nf}B_{o}V^{2}=0. \end{array}$$

Introduce the following nondimensional parameters. Eqs. (11) and (12), with the boundary conditions become, work done due to deformation and Joule heating in a nondimensional form is given as

(14) $$\begin{array}{c} u=\bar{u}U,\\ \bar{T}=\frac{T-T_{1}}{T_{2}-T_{1}}, \end{array}$$

(15) $$\begin{array}{c} \frac{d^{2}u}{dy^{2}}+6\beta {\left(1-\psi \right)}^{2.5}{\left(\frac{du}{dy}\right)}^{2}\frac{d^{2}u}{dy^{2}}-{\left(1-\psi \right)}^{2.5}m_{2}\text{Mu}+{\left(1-\psi \right)}^{2.5}m_{3}K=0, \end{array}$$

with boundary conditions

(16) $$\begin{array}{c} u\left(-1\right)=0, \end{array}$$

(17) $$\begin{array}{c} \left(1+\frac{4N}{3m_{1}}\right)\frac{d^{2}\theta }{dy^{2}}+\frac{B_{r}}{m_{1}{\left(1-\psi \right)}^{2.5}}{\left(\frac{du}{dy}\right)}^{2}+\frac{2\beta B_{r}}{m_{1}}{\left(\frac{du}{dy}\right)}^{4}+\frac{m_{2}B_{r}}{m_{1}}{\text{Mu}}^{2}=0, \end{array}$$

with boundary conditions

(18) $$\begin{array}{c} \theta \left(-1\right)=0,\\ \theta \left(1\right)=1, \end{array}$$

where *β*=(*U*/*H*)^2^*β*_2_+*β*_3_/*μ*_*f*_ is a third-grade fluid parameter, *K*=*ρ*_*f*_*gH*^2^/*Uμ*_*f*_sin  *ϕ* is a gravitational parameter, *M*=*B*_0_^2^*σ*_*f*_*H*^2^/*μ*_*f*_ is a magnetic parameter, *B*_*r*_=*U*^2^*μ*_*f*_/*k*_*f*_Δ*T* is the Brinkman number, and *N*=4*σ*^*∗*^*T*_*∞*_^3^/*k*_*f*_(*ρc*_*p*_)_*f*_*k*^*∗*^ is the thermal radiation.

The article "Numerical Simulation of MHD Couette Flow of a Fuzzy Nanofluid through an Inclined Channel with Thermal Radiation Effect" was published in 2021. Journal: Comput Intell Neurosci.

Here, *ρ*_*nf*_, *μ*_*nf*_, *k*_*nf*_, (*ρC*_*p*_)_*nf*_, *σ*_*f*_,  and *ψ* denote the density, viscosity, thermal conductivity, specific heat, electrical conductivity, and nanoparticles' volume fraction of nanofluids, respectively [29, 32].

(19) $$\begin{array}{c} m_{3}=\rho_{nf}=\left[\left(1-\psi \right)+\psi \frac{\rho_{s_{3}}}{\rho_{f}}\right]\rho_{f},\\ \mu_{nf}=\mu_{f}{\left(1-\psi \right)}^{-2.5},\\ m={\left(\rho c_{p}\right)}_{nf}=\left[\left(1-\psi \right){\left(\rho c_{p}\right)}_{f}+\psi {\left(\rho c_{p}\right)}_{s_{5}}\right],\\ m_{1}=\frac{k_{nf}}{k_{f}}=\frac{2k_{f}+2\psi_{1}\left(k_{s_{1}}-k_{f}\right)+k_{s_{1}}}{2k_{f}-\psi_{1}\left(k_{s_{1}}-k_{f}\right)+k_{s_{1}}},\\ m_{2}=\frac{\sigma_{nf}}{\sigma_{f}}=1+\frac{3\left(\sigma_{s_{4}}-\sigma_{f}\right)\psi }{\left(\sigma_{s_{4}}+2\sigma_{f}\right)-\left(\sigma_{s_{4}}-\sigma_{f}\right)\psi }. \end{array}$$

The properties of the base fluid and nanoparticles are listed in Table 1.

### 3.1. Formulation of the Crisp Problem into the Fuzzy Problem Using FDEs

The velocity and temperature are affected by a small change in the value of the volume fraction of nanoparticles. Some researchers take the volume fraction of nanoparticles in the range [0.01–0.04], so the point is that the flow of fluid just depends on these values. Then, uncertainty arises due to the fixed crisp values of the volume fraction of nanoparticles. So, it is better to handle a difficult problem in a fuzzy environment by taking volume fraction as the FN.

The article "Numerical Simulation of MHD Couette Flow of a Fuzzy Nanofluid through an Inclined Channel with Thermal Radiation Effect" was published in 2021. Journal: Comput Intell Neurosci.

For the fuzzy form, the governing coupled differential equations (15)–(18) can be written as

(20) $$\begin{array}{c} \frac{d^{2}\bar{u}\left(y,\;\alpha \right)}{dy^{2}}+6\beta {\left(1-\bar{\psi }\right)}^{2.5}{\left(\frac{d\bar{u}\left(y,\alpha \right)}{dy}\right)}^{2}\frac{d^{2}\bar{u}\left(y,\alpha \right)}{dy^{2}}-{\left(1-\bar{\psi }\right)}^{2.5}m_{2}M\bar{u}\left(y,\alpha \right)+{\left(1-\bar{\psi }\right)}^{2.5}m_{3}K=0, \end{array}$$

(21) $$\begin{array}{c} \left(1+\frac{4N}{3m_{1}}\right)\frac{d^{2}\bar{\theta }\left(y,\;\alpha \right)}{dy^{2}}+\frac{B_{r}}{m_{1}{\left(1-\bar{\psi }\right)}^{2.5}}{\left(\frac{d\bar{u}\left(y,\alpha \right)}{dy}\right)}^{2}+\frac{2\beta B_{r}}{m_{1}}{\left(\frac{d\bar{u}\left(y,\alpha \right)}{dy}\right)}^{4}+\frac{m_{2}B_{r}}{m_{1}}M{\bar{u}}^{2}\left(y,\alpha \right)=0, \end{array}$$

with boundary conditions

(22) $$\begin{array}{c} \bar{u}\left(y,\alpha \right)=0,\bar{\theta }\left(y,\alpha \right)=0\text{ at }y=-1,\\ \bar{u}\left(y,\alpha \right)=1,\bar{\theta }\left(y,\alpha \right)=1\text{ at }y=1. \end{array}$$

For the fuzzy solution, equations (15)–(18) can be converted into FDEs using the *α*‐cut approach. So, according to Definitions 4 and 5, we have

(23) $$\begin{array}{c} \frac{d^{2}}{dy^{2}}\left(u_{1}\left(y,\alpha \right),u_{2}\left(y,\alpha \right)\right)+6\beta {\left(1-\bar{\psi }\right)}^{2.5}{\left(\frac{d}{dy}\left(u_{1}\left(y,\alpha \right),u_{2}\left(y,\alpha \right)\right)\right)}^{2}\frac{d^{2}}{dy^{2}}\left(u_{1}\left(y,\alpha \right),u_{2}\left(y,\alpha \right)\right)\\ -{\left(1-\bar{\psi }\right)}^{2.5}m_{2}M\left(u_{1}\left(y,\alpha \right),u_{2}\left(y,\alpha \right)\right)+{\left(1-\bar{\psi }\right)}^{2.5}m_{3}K=0, \end{array}$$

(24) $$\begin{array}{c} \left(1+\frac{4N}{3m_{1}}\right)\frac{d^{2}}{dy^{2}}\left(\theta_{1}\left(y,\alpha \right),\theta_{2}\left(y,\alpha \right)\right)+\frac{B_{r}}{m_{1}{\left(1-\bar{\psi }\right)}^{2.5}}{\left(\frac{d}{dy}\left(u_{1}\left(y,\alpha \right),u_{2}\left(y,\alpha \right)\right)\right)}^{2}+\frac{2\beta B_{r}}{m_{1}}{\left(\frac{d}{dy}\left(u_{1}\left(y,\alpha \right),u_{2}\left(y,\alpha \right)\right)\right)}^{4}\\ +\frac{m_{2}B_{r}}{m_{1}}M\left(u_{1}\left(y,\alpha \right),u_{2}\left(y,\alpha \right)\right)=0, \end{array}$$

with boundary conditions

(25) $$\begin{array}{c} \left(u_{1}\left(y,\alpha \right),u_{2}\left(y,\alpha \right)\right)=\left(0,0\right),\left(\theta_{1}\left(y,\alpha \right),\theta_{2}\left(y,\alpha \right)\right)=\left(0,0\right)\text{ at }y=-1,\\ \left(u_{1}\left(y,\alpha \right),u_{2}\left(y,\alpha \right)\right)=\left(1,1\right),\left(\theta_{1}\left(y,\alpha \right),\theta_{2}\left(y,\alpha \right)\right)=\left(1,1\right)\text{ at }y=1, \end{array}$$

where “^___^” stands for the fuzzy form and fuzzy velocity profile is $\bar{u}\left(y,\alpha \right)=\left[u_{1}\left(y,\alpha \right),u_{2}\left(y,\alpha \right)\right],\;0\leq \alpha \leq 1$. Here, *u*_1_(*y*, *α*) is the lower bound and *u*_2_(*y*, *α*) the upper bound of fuzzy velocity profiles. Similarly, the fuzzy temperature profiles are $\bar{\theta }\left(y,\alpha \right)=\left[\theta_{1}\left(y,\alpha \right),\theta_{2}\left(y,\alpha \right)\right],\;0\leq \alpha \leq 1$.

The article "Numerical Simulation of MHD Couette Flow of a Fuzzy Nanofluid through an Inclined Channel with Thermal Radiation Effect" was published in 2021. Journal: Comput Intell Neurosci.

The crisp values and TFNs of these FNs are listed in Table 2. The TFN defined the variation of the FN at each *α*‐cut. The TFNs are used to describe the triangular membership functions of the FNs which range from 0 to 1; see Figure 1. The investigated ranges are generally used to build up the said problem.

Now we proposed a numerical method bvp4c to solve crisp differential equations and FDEs. It is a Lobatto IIIa formula with three stages based on the finite-difference algorithm. It has a collocation polynomial, and in [*a*, *b*], the collocation formula yields a sixth-order accurate uniform C1 continuous solution. For error control and mesh selection, the continuous solution residual is employed. Further solvers, such as NDSOLVE, HPM, HAM, and ADM, and many other similar approaches are less consistent than bvp4c.

We transformed the governing ODEs to the system of the first order as follows.

Let

(26) $$\begin{array}{c} u\left(y\right)=w\left(1\right)\\ u^{\prime \prime }\left(y\right)=w^{\prime \prime }\left(1\right)=w^{\prime }\left(2\right), \end{array}$$

(27) $$\begin{array}{c} w^{\prime }\left(2\right)=\frac{{\left(1-\psi_{1}\right)}^{2.5}m_{2}Mw\left(1\right)-{\left(1-\psi_{1}\right)}^{2.5}m_{3}K}{1+6\beta {\left(1-\psi_{1}\right)}^{2.5}{\left(w\left(2\right)\right)}^{2}}, \end{array}$$

(28) $$\begin{array}{c} \theta \left(y\right)=w\left(3\right),\\ \theta^{\prime }\left(y\right)=w^{\prime }\left(3\right)=w\left(4\right),\\ \theta^{\prime \prime }\left(y\right)=w^{\prime }\left(4\right), \end{array}$$

(29) $$\begin{array}{c} w^{\prime }\left(4\right)=\frac{-3}{3m_{1}+4N}\left[\frac{Br{\left(w\left(2\right)\right)}^{2}}{{\left(1-\psi \right)}^{2.5}}+2\beta Br{\left(w\left(2\right)\right)}^{4}+m_{1}MBr{\left(w\left(1\right)\right)}^{2}\right]. \end{array}$$

Boundary conditions are

(30) $$\begin{array}{c} w_{a}\left(1\right)=0,\\ w_{b}\left(1\right)=1,\\ w_{a}\left(3\right)=0,\\ w_{b}\left(3\right)=1. \end{array}$$

To find the solution of Eqs. (24) to (28), a code in MATLAB software for bvp4c method is constructed.

The article "Numerical Simulation of MHD Couette Flow of a Fuzzy Nanofluid through an Inclined Channel with Thermal Radiation Effect" was published in 2021. Journal: Comput Intell Neurosci.

## 4. Results and Discussion

In this section, pure water (H_2_O) is chosen as a base fluid, and SWCNT and MWCNT are nanoparticles added into the base fluid to enhance the heat transfer rate between two heated inclined parallel plates. The numerical solutions of governing coupled nonlinear differential equations are achieved through numerical technique bvp4c. The effect of crisp thermophysical parameters, such as nanoparticle volume fraction *ψ*, gravitational parameter *K*, magnetic parameter *M*, Brinkman number *Br*, and nondimensionless non-Newtonian viscosity *β*, on velocity and temperature profiles is drawn in Figures 3–8.

Tables 3 and 4 show the comparison of velocity and temperature fields for different values of *β* [10, 11] when *K*=1, *Br*=5, *M*=5, *N*=0,  and *ψ*=0. The validation of our results of the present study was found to be in excellent agreement.

Figure 3 demonstrates the impact of *β* on velocity and temperature profiles when other parameters are fixed. It is seen that the velocity and temperature of the nanofluid increase with increasing the values of *β* because of the increase in the boundary layer thickness.  Figure 4 displays the influence of gravitational parameter *K* on velocity and temperature profiles when other physical parameters are fixed. It is noticed that the velocity and temperature of the nanofluid rise rapidly in the center of the inclined plates with increasing the values of *K.* The reason is that when *K* increases, the upper plate movement expands the nanofluid velocity, which strengthens Joule dissipation; thereby, the rate of heat transfer is enhanced. The effect of *M* on the velocity and temperature profile is seen in Figure 5. When the value of *M* is increased, the velocity drops due to the Lorentz forces, but the temperature profile rises. The rate at which the nanofluid flow declines is less noticeable from the lower plate to the higher plate. Physically, when the magnetic parameter rises, the rate of nanofluid flow near the moving upper plate is significantly reduced compared to the stationary lower plate. Also, it is noticed that increases in the magnetic parameter cause an increase in Joule heating, which raises the heat transfer rate.  Figure 6 visualizes the effect of *N* on the nanofluid of the temperature profile. As depicted, it is seen that the temperature profile performs a decreasing function with increasing *N*, therefore, representing a damping impact on the heat transfer performance and nanofluid flow. The effect of the viscous dissipation parameter *Br* on the temperature profile is demonstrated in Figure 7. It is observed that the temperature of the nanofluid increases with increasing the values of *Br*. The physical meaning of *Br* is when *Br* increases, the dissipation of heat in the boundary layer region increases, so the flow of the nanofluid is enhanced, and the heat transfer rate grows.

The article "Numerical Simulation of MHD Couette Flow of a Fuzzy Nanofluid through an Inclined Channel with Thermal Radiation Effect" was published in 2021. Journal: Comput Intell Neurosci.

The effect of *ψ* via the velocity profile of nanomaterials SWCNT and MWCNT is shown in Figure 8(a). When *ψ* increases, the velocity of the nanofluid decreases. The velocity of the regular fluid is maximum at *ψ*=0, which means that, by increasing the nanofluid volume fraction, it becomes denser. Physically, it means that the boundary layer of nanofluids is thicker than regular fluids; consequently, the velocity shows a decreasing behavior with increasing values of *ψ*. The effect of *ψ* on the temperature profile of nanomaterials SWCNT and MWCNT is depicted in Figure 8(b). It can be seen that the temperature profiles increase with an increase in *ψ*. Physically, this is true because of the thicker thermal boundary layer which increases the heat transfer.

Now, we discuss the nanoparticles' volume fraction of the SWCNT and MWCNT in a fuzzy environment. The governing equations of momentum and energy are converted into FDEs; then, the bvp4c scheme is employed for the numerical solution. The nanoparticle volume fraction *ψ* is taken as TFN (see Table 2). Moreover, we utilized the *α*-cut approach (0≤α≤1) to analyze the uncertainty. Then, the velocity and temperature profiles are said to be fuzzy. The *α*‐cut controls the fuzzy terms, for instance, if *α*‐cut=0, it will cover the whole interval of nanoparticles' volume fraction; that is, *ψ*=[0,0.2]. *α*-cut increases as (0.05 to 0.95) the width of lower and upper bounds of fuzzy velocity or temperature profiles decreases. When *α*-cut = 1, then the lower and upper bounds of fuzzy velocity or temperature profiles are coherent with each other, so they provide a crisp result. It is important to note that if the width between lower and upper bounds of the velocity or temperature profile is less, the uncertainty is less. The fuzzy velocity and temperature profiles are plotted in Figures 9 and 10 for some particular values of *α*‐cut, (*α*=0,  0.3,  0.6,  and 1). The triangular membership functions are depicted in Figures 11 and 12 for different values of *y*.

Figures 9 and 10 show the nanoparticles' volume fraction of SWCNTs and MWCNTs taken as the TFN (see in Table 1); then, the fuzzy velocity and temperature profiles are controlled by *α*‐cut (*α* ∈ [0,1]). Figures 9(a) and 10(a) describe the effect of the *α*‐cut on fuzzy velocity profile $\bar{u}\left(y,\alpha \right)$ for the volume fraction of SWCNTs and MWCNTs which are TFNs, respectively. It is seen that *α* significantly affects the fuzzy velocity profile of the regular fluid and nanofluid. The lower bound of the velocity profile shows the regular fluid, and the upper bound of the velocity profile displays the nanofluid at *α*=0. Physically, it means that, at *α*=0, the thermal boundary layer of *u*_1_(*y*, *α*) is thinner, and the thermal boundary layer of *u*_2_(*y*, *α*) is denser. The velocity of a regular fluid is maximum compared to the velocity of the nanofluid for different values of *α*. When *α*‐cut increases, the width between *u*_1_(*y*, *α*) and *u*_2_(*y*, *α*) decreases, and at *α*‐cut=1, they coherent with one another which is a real flow of the nanofluid. It is noted that the width between *u*_1_(*y*, *α*) and *u*_2_(*y*, *α*) is very less, so the uncertainty is less.

The article "Numerical Simulation of MHD Couette Flow of a Fuzzy Nanofluid through an Inclined Channel with Thermal Radiation Effect" was published in 2021. Journal: Comput Intell Neurosci.

The effect of the *α*‐cut on temperature profile $\bar{\theta }\left(y,\;\alpha \right)$ is represented in Figures 9(b) and 10(b) for the fuzzy volume fraction of SWCNTs and MWCNTs, respectively. The lower bound of the temperature profile shows the regular fluid, and the upper bound of the temperature profile shows the nanofluid at *α*=0. Physically, it means that, at *α*=0, the thermal boundary layer of *θ*_1_(*y*,  *α*) is denser, and the thermal boundary layer of *θ*_2_(*y*,  *α*) is thinner. Momentum and thermal boundary layers show opposite behavior at *α*=0, which shows that the heat transfer is maximum. When *α*‐cut increases, the width between *θ*_1_(*y*,  *α*) and *θ*_2_(*y*,  *α*) decreases, and at *α*‐cut=1, they coherent with one another which is the real flow of the nanofluid. It is noted that the width between *θ*_1_(*y*,  *α*) and *θ*_2_(*y*,  *α*) is very less, so the uncertainty is less.

The comparison of SWCNTs and MWCNTs through fuzzy plots for various values of *y* is depicted in Figures 11 and 12. The volume fraction of SWCNTs and MWCNTs is the TFN. Figures 11 and 12 represent the fuzzy plots of fuzzy velocity and temperature profiles for different values of *y*. The fuzzy velocity of SWCNTs is greater than the fuzzy velocity of MWCNTs. Physically, it is correct because the density of SWCNTs is less than the density of MWCNTs. Comparing for the fuzzy temperature distribution, SWCNTs have greater thermal conductivity than MWCNTs but less density. So, SWCNTs bear more heat than MWCNTs, and in this study, we suggest that SWCNTs are better for the enhanced heat transfer as compared to MWCNTs. Also, the SWCNTs show better behavior as compared to MWCNTs because of their less width according to the membership function.

## 5. Conclusion

In this study, the effect of CNTs on MHD Couette flow via an inclined channel in a fuzzy environment is reported. The SWCNTs and MCNTs are nanoparticles, while pure water is the base fluid. The effects of Brinkman number (*B*_*r*_), magnetic parameter (*M*), the volume fraction of nanoparticles (*ψ*), viscosity (*β*), thermal radiation (*N*), and gravitational parameter (*K*) are considered. The impact of different parameters on heat transfer, velocity, and temperature profiles is analyzed. For mathematical computation, bvp4c is used, and the present results are found to be in excellent agreement as compared to existing results. The governing nonlinear DEs are converted into FDEs; then, the numerical technique bvp4c employed. The volume fraction of nanoparticles is considered as TFNs through *α*‐cut(0 ≤ *α* ≤ 1), and the fuzziness is controlled. Some of the important and convenient achieved results are as follows:

- The velocity and temperature profiles increase when the gravitation parameter (*K*) and fluid parameter (*β*) increase.
- The velocity profile decreases when a magnetic parameter (*M*) increases, and the temperature profile increases near the boundary layer.
- The temperature profile decreases when the thermal radiation parameter (*N*) increases due to heat transfer. The temperature profile increases with an increase in the Brinkman number (*Br*).
- The temperature profile increases and the velocity profile decreases when the volume fractions of SWCNTs and MWCNTs increase.
- The comparison of SWCNTs and MWCNTs shows that SWCNTs have a better heat transfer rate as compared to MWCNTs. Also, the comparison of SWCNTs and MWCNTs is examined through triangular membership plots of fuzzy velocity and temperature profiles, which shows that the width of MWCNTs is greater than that of SWCNTs.
- The results indicate that the crisp solution is always in-between the upper and lower solutions when *α*‐cut increases from 0 to 1. The lower solution shows the minimum flow of the fluid (regular fluid), and the upper solution shows the maximum flow of the nanofluid when *α*‐cut=0.
- In future works, one can use other fuzzy numbers to solve the heat transfer problems.

The article "Numerical Simulation of MHD Couette Flow of a Fuzzy Nanofluid through an Inclined Channel with Thermal Radiation Effect" was published in 2021. Journal: Comput Intell Neurosci.

## Figures and Tables

**Figure 1:** Membership functions of a TFN.

**Figure 2:** Geometry of the problem.

**Figure 3:** Influence of *β* on *u*(*y*) and *θ*(*y*).

**Figure 4:** Influence of *K* on *u*(*y*) and *θ*(*y*).

**Figure 5:** Influence of *M* on *u*(*y*) and *θ*(*y*).

**Figure 6:** Influence of *N* on *θ*(*y*).

**Figure 7:** Influence of *Br* on *θ*(*y*).

**Figure 8:** Influence of *ψ* on *u*(*y*) and *θ*(*y*).

**Figure 9:** Effect of the fuzzy volume fraction of the nanofluid (SWCNT) on $\bar{u}\left(y,\alpha \right)\text{ and }\bar{\theta }\left(y,\alpha \right)$.

**Figure 10:** Effect of the fuzzy volume fraction of the nanofluid (MWCNT) on $\bar{u}\left(y,\alpha \right)\text{ and }\bar{\theta }\left(y,\alpha \right)$.

**Figure 11:** Effects of the TFN volume fraction of the SWCNT and MWCNT on $\bar{u}\left(y,\alpha \right)$. (a) At *y* = −0.25. (b) At *y* = 0.25. (c) At *y* = −0.75. (d) At *y* = 0.75.

**Figure 12:** Effects of the TFN volume fraction of the SWCNT and MWCNT on $\bar{\theta }\left(y,a\right)$ (a) At *y* = −0.25. (b) At *y* = 0.25. (c) At *y* = −0.75. (d) At *y* = 0.75.

**Table 1:** Thermophysical properties of the base fluid and nanoparticles.

Materials	*ρ*(kg/m^3^)	*Cρ*(J/kgK)	*k*(W/m)	*σ*(s/m)
Pure water	997.1	4179.0	0.6130	0.05
SWCNTs	2600.0	425.0	6600.0	21
MWCNTs	1600.0	796.0	3000.0	44

**Table 2:** TFNs of fuzzy nanoparticles of volume fraction.

Fuzzy number	Crisp value	TFN	*α*‐cut approach
*ψ*	0.01–0.04	[0, 0.1, 0.2]	[0+0.1*α*, 0.2 − 0.1*α*], *α* ∈ [0,1]

**Table 3:** Comparison of numerical results with analytical results for the velocity of Couette flow when *K*=1, *Br*=5, *M*=5, *N*=0,  and *ψ*=0.

*β*=0.001				*β*=0.1		
*Y*	PM [10]	ADM [11]	Present results (bvp4c)	PM [10]	ADM [11]	Present results (bvp4c)
−1	0	0	0	0	0	0
−0.8	0.080599	0.080571	0.080607	0.0.81260	0.081425	0.083115
−0.6	0.136936	0.136935	0.136939	0.140203	0.143142	0.142375
−0.4	0.180453	0.180451	0.180449	0.187494	0.187499	0.189643
−0.2	0.219997	0.21999	0.219984	0.232351	0.234952	0.233923
0	0.263605	0.263606	0.263602	0.283677	0.283699	0.283364
0.2	0.320143	0.320145	0.320104	0.351506	0.355152	0.347445
0.4	0.401095	0.401099	0.400987	0.448301	0.450123	0.436373
0.6	0.522872	0.522972	0.522653	0.578833	0.578958	0.563876
0.8	0.710055	0.721005	0.709739	0.753411	0.756252	0.746170
1	1	1	0.999997	1	1	1

**Table 4:** Comparison of numerical results with analytical results for the temperature of Couette flow when *K*=1, *Br*=5, *M*=5, *N*=0,  and *ψ*=0.

*β*=0.001				*β*=0.1		
*Y*	PM [10]	ADM [11]	Present results (bvp4c)	PM [10]	ADM [11]	Present results (bvp4c)
−1	0	0	0	0	0	0
−0.8	1.22328	1.25252	0.533675	1.402449	1.52425	0.596488
−0.6	2.34181	2.42512	1.037249	2.404120	2.50214	1.159899
−0.4	3.31125	3.42523	1.509760	3.151470	3.12542	1.688806
−0.2	4.09503	4.10295	1.941188	3.982890	3.89898	2.171262
0	4.65215	4.56522	2.315419	4.776961	4.65824	2.587627
0.2	4.91100	5.00252	2.606950	5.081522	5.00252	2.906360
0.4	4.81112	4.91252	2.770656	4.783381	4.78588	3.072202
0.6	4.33810	4.45210	2.718227	4.162820	4.21500	2.980832
0.8	3.17165	3.01255	2.264215	3.194671	3.20125	2.426644
1	1	1	1	1	1	1

## Data Availability

No data were used to support this study.

## Abbreviations

$\bar{x},\;\bar{y}$: Cartesian coordinates
*u*: Normal component of the flow
*T*: Transpose of the matrix
*θ* (*y*): Dimensionless temperature
*T*_1_, *T*_2_: Reference and ambient temperatures
*M*: Magnetic parameter
*Br*: Brinkman number
*β*: Third-grade fluid parameter
*P*: Pressure
$\hat{S}$: Cauchy stress tensor
*α*_1_, *α*_2_, *β*_1_, *β*_2_, and *β*_3_: Material constants
*μ*_*m*_: Magnetic permeability
*μ*: Coefficient of viscosity
$\bar{\theta }\left(y,\alpha \right)$: Fuzzy temperature profile
*σ* ^*∗*^: Stefan–Boltzmann constant
*k* ^*∗*^: Absorption coefficient
*N*: Thermal radiation
*ρ*_*nf*_: Density of the nanofluid
*μ*_*nf*_: Viscosity of the nanofluid
(*ρC*_*p*_)_*nf*_: Specific heat of the nanofluid
*ψ*: Nanoparticles' volume fraction
*θ*_1_(*y*, *α*): Lower fuzzy temperature profile
*θ*_2_(*y*, *α*): Upper fuzzy temperature profile
*d/dt*: Material derivative
*δ*: Electrical conductivity
*K*: Gravitational parameter
*ρ*: Density of the fluid
*α*: Level or cut technique
FDE: Fuzzy differential equation
$\mu_{\bar{U}}\left(x\right)$: Membership function
$\bar{u}\left(y,\;\alpha \right)$: Fuzzy velocity profile
*u*_1_(*y*, *α*): Lower fuzzy velocity profile
*u*_2_(*y*, *α*): Upper fuzzy velocity profile
TFN: Triangular fuzzy number
*B*: Total magnetic field
*f*: External body force
*A*_*n*_: Rivlin–Ericksen tensors
*A*_∘_: Identity tensor
*H*: Distance between two plates
*k*_*nf*_: Thermal conductivity of the nanofluid
*σ*_*f*_: Electrical conductivity of the nanofluid.
